RETRACTED

# Innovating a Practical Teaching Base of Landscape Architecture Major Based on the Campus Environment: A Case Study of Xuzhou University of Technology (China)

**DOI:** 10.1155/2022/6209454

**Published:** 2022-06-20

**Authors:** Xuehong Tan, Pin Liu, Nan Nan, Yunle Peng

**Affiliations:** ^1^School of Environmental Engineering, Xuzhou University of Technology, Xuzhou 221008, China; ^2^School of Arts, Xuzhou University of Technology, Xuzhou 221008, China

## Abstract

Xuzhou University of Technology is a local newly established applied undergraduate university. The construction of a practical teaching base of landscape architecture majors was faced with the problems of short construction time and lack of funds. The feasibility, necessity, process, and achievements of the construction of the practical teaching base of landscape architecture majors based on the campus environment were studied. The guiding ideology of the campus practical teaching base for landscape architecture majors in applied undergraduate universities was put forward and the construction mode of “four in one” of practical teaching bases was discussed. The campus practical teaching base for landscape architecture majors was built and “four-stage” progressive training and teaching activities were carried out in Xuzhou University of Technology. The effective combination of the landscape architecture professional practical teaching base and the logistics resources was realized. The combination of the logistics resources and professional construction of the university was carried out as a beneficial exploration in this paper. The achievements of practical teaching base construction were mainly reflected in the improvement of the quality of talent cultivation, the beautification of campus environment, and the enhancement of teachers practical ability.

## 1. Introduction

According to the statistics of China landscape architecture education conference in 2014, more than 220 colleges and universities in China had opened undergraduate majors of landscape architecture, gardening, and related majors, and more than 50,000 students of related majors at all levels were enrolled every year [1,2]. As we all know, landscape architecture was a highly practical subject; the study of landscape architecture students should not be limited to classroom theoretical teaching and practical teaching was an important link to cultivate students' application ability and innovation ability; the practical teaching base was the main place to cultivate landscape architecture students' practical ability and innovation ability [3,4]. However, many newly built local undergraduate colleges were unable to build practical teaching bases for landscape architecture majors as compared with those key universities due to the short construction time and lack of funds, which directly affected the quality of students' training.

RETRACTED

Xuzhou University of Technology (hereafter abbreviated as our university) was a local established applied undergraduate university, and our university closely adhered to the mainline of local and application-oriented education, practiced the concept of “big application view, big engineering view, big life view, and big culture view,” and realized the road of innovative development of the university [5]. In order to achieve the goal of cultivating senior application-oriented talents with solid theoretical knowledge and strong practical ability in landscape architecture majors of our university, it was necessary to build a practical teaching base with strong practicability to ensure the quality of talent's cultivation. In order to save money and shorten the construction time, our university put forward the suggestion of constructing a practical teaching base for landscape architecture major relying on the campus environment. The facts proved that the practical teaching base of landscape architecture majors established on the campus environment of our university had realized the combination of theory teaching and practice and the unity of practice and production; it had strengthened the enthusiasm of students in learning, stimulated their creativity and innovation, and narrowed the distance between teaching and production.

Therefore, the landscape architecture major of our university realized the smooth integration of students from campus practice to off-campus work and shortened the employment adaptation period of graduates [6].

## 2. Theoretical Exploration

### 2.1. Guiding Ideas of the Building Practical Teaching Base of Landscape Architecture Major on the Campus

Practical teaching referred to the practical activities carried out around teaching activities and students' personal experience, and the practical teaching base was the material basis for the development of practical teaching [7]. Our university began to recruit landscape architecture majors in 2015. There are 312 students of this major in our school at present. The major had a large number of practical courses, such as landscape botany practice, landscape architecture design practice, landscape planning and design practice, landscape engineering practice, plant landscape design practice, cognitive practice, model making, comprehensive practice, graduation design, graduation practice, etc. With the revision of the 2019 version of the talent cultivating program, the number of teaching hours of practical training had been increased. Practical teaching was 65.5 credits, accounting for 40.18% of the total credits in the talent cultivating program for landscape architecture majors. A large number of practical courses needed to be completed in the practical teaching base in order to master the practical operation skills in the field of landscape architecture and the students could get rid of the monotonous “cramming” classroom.

RETRACTED

Therefore, the guiding ideology of the construction of the practical teaching base for landscape architecture major in our university was that the talent cultivating program combined theory with practice, aimed at cultivating students' practical ability and innovative consciousness, adhered to combine the construction, transformation, and maintenance of the campus environment with students' practical training courses. The practical teaching base of the campus environment should become a real practice environment in the garden industry and an open practice teaching base integrating teaching, production, and scientific research.

### 2.2. The Mode of “Four in One” Practical Teaching Base Construction

Relying on the campus environment, under the guidance of the leaders of university, the college and the logistics department cooperated to set up an open practical teaching base on the campus, which could realize the “four-in-one” function of practical teaching, technological innovation, construction of professional culture, and beautification of campus environment (Figure 1) and the practical teaching base had strong practicability. The construction of the practical teaching base adhered to the three-dimensional principle of “landscape of the practical environment, teaching of the campus environment, and humanistic culture of the campus environment.” All kinds of plants and landscape on campus not only served for professional teaching, reflected professional cultural connotation, provided the place for curriculum reform and the source of innovation but also had the function of beautifying the environment. Students on campus could recognize the main elements of landscape architecture, subtly cultivate the perception and experience of beauty, feel the sense of professional well-being, and stimulate interest in learning and professional love.

The model of “four-in-one” practical teaching base construction realized the effective cooperation of various departments in the university, improved the management efficiency of the campus environment, and saved the construction cost of the practical teaching base, so it was of great significance.

## 3. The Practice of Practical Teaching Base Construction

### 3.1. Establishing a Practical Teaching Base for Landscape Architecture Major on the Campus

The traditional form of practical training and the practical teaching system in colleges and universities was mainly based on teacher demonstration and the students in a passive position. Therefore, it was difficult for students to have interest in practical training and practical teaching, which restricted the cultivation of students' practical ability [8,9]. As a local applied undergraduate university, our university had already realized this point and the university leaders broke through the thinking barrier and innovated boldly. Under the leadership of the university, the college of environmental engineering and the logistics office had successively negotiated and signed a cooperation agreement in April 2015 based on the principle of resource sharing, complementary advantages, and mutual benefit. According to the agreement, the college of environmental engineering contracted the 110,000 square meters of green maintenance and landscape renovation projects on the campus and established a campus practical teaching base of landscape architecture major with the logistics office.

RETRACTED

After nearly four years of operation, the base not only provided the course practice of landscape dendrology, floriculture, lawn science, garden plant cultivation and maintenance, landscape planning and design, plant planning and design, landscape engineering and other courses but also became the place of graduation practice, second classroom, scientific and technological innovation for some students, as well as the place for the display of landscape architecture professional culture. At the same time, the campus was beautified, the funds were saved, and the real design and construction environment was provided for students through the projects of flower planting in tree pools, *Prunus mume* forest transformation and *Cedrus deodara* forest transformation.

### 3.2. Realizing the Effective Combination of the Practical Teaching Base of Landscape Architecture Major and Logistics Resources

Campus greening maintenance and landscape transformation spent a lot of manpower, financial, and material resources every year. In order to achieve the dual objectives of mutual benefit and students' practical ability training, and to ensure the sustainability and practicability of the practical teaching base, the college of environmental engineering (Landscape architecture major belonged to the college of environmental engineering) and the logistics office signed a long-term internship cooperation agreement to build a practical teaching base of landscape architecture majors. Under the guidance of the university, leadership and the assistance of the equipment office, the finance office, the dean's office, and the student affairs office, the basic mode of co-construction of the practical teaching base between college and logistics was established (Figure 2), which formed the relationship of interdependence and in-depth cooperation.

RETRACTED

The establishment of the campus environment practical teaching base saved the school's expenses, where the teachers and students built the campus environment as masters. The teachers and students had a sense of belonging and a stronger responsibility, so they had targeted the landscape transformation of the campus environment and could create a suitable space environment for the teachers and students of the university to work, study, and live. On the other hand, the campus practical teaching base of landscape architecture majors broke the traditional single and laboratory-limited mode of the practical teaching base of landscape architecture majors, made full use of the effective logistics resources, and maximized its advantages. Therefore, the establishment of a practical teaching base of landscape architecture major based on the campus environment was an effective combination of professional teaching and logistics resources to achieve a win-win goal.

In the management of the practical teaching base, the system of co-management of college teachers and logistics personnel was explored. The college and logistics office jointly set up a leadership group to formulate a practical teaching base management program and a practical teaching model for students. The landscape architecture teachers and logistics greening team members were responsible for the content and arrangement of students' practice. The college and the logistics office selected teachers to jointly guide students' practical training (Figure 3).

### 3.3. Realizing the “Four-Stage” Progressive Practical Teaching Chain

The boring theoretical knowledge should be combined with practical teaching to understand and deepen the theoretical knowledge in practice and to develop students' practical ability. Students' consciousness and ability of innovation and entrepreneurship should be cultivated throughout the whole teaching process [10,11]. According to students' cognitive order and the needs of campus environment construction, transformation, and beautification, a “four-stage” progressive practical teaching chain for landscape architecture majors had formed and each stage could be completed in the campus practical teaching base.

The “four-stage” referred to the basic practical ability training stage, the professional core skill training stage, the comprehensive application ability training stage, and the innovation and entrepreneurship capacity training stage of the students. The training courses and time schedules of the “four-stage” corresponding ability are shown in Table 1. The “four-stage” training chain was progressively carried out in terms of students' practical ability training, and there were overlaps and intersections in the time schedule of the training courses. For example, the cultivation of students' innovation and entrepreneurship ability had been carried out since the second year of the course. Students were encouraged to participate in teachers' scientific research and to declare innovative and entrepreneurship training projects; the cultivation of students' innovation and entrepreneurship ability had continued until graduation.

RETRACTED

In the basic practical ability training stage, students' main practical courses included cognitive practice, art sketch, surveying practice, and landscape botany practice, which were arranged in semesters 1–4. In the professional core skills training phase, students' main practical courses included landscape architecture design practice, landscape planning and design practice, landscape engineering practice, and plant landscape design practice, which were arranged in semesters 4–6. In the comprehensive application ability training stage, students' main practical courses included comprehensive practice and graduation design, which were arranged in semesters 6–8. In the innovation and entrepreneurship capacity training stage, students' main practical courses included innovation and entrepreneurship quality education for university students, graduation practice, innovation, and entrepreneurship competition, which were arranged in semesters 2–8.

## 4. Achievements of the Practical Teaching Base

### 4.1. Significant Improvement in the Quality of Talent Cultivation

Since the foundation of the base in 2015, there were more than 200 class hours practical training every year in the base, 30 students had graduation practice in the campus practical teaching base, and 6 students chose the theme of graduation design as campus landscape transformation. Two competetions: a “landscape design competition” (Figure 4) and a “plant pruning competition” (Figure 5) were held in the campus practical teaching base. Through the establishment of a green protection team and campus landscape renovation program bidding activities, students' practical ability and teamwork awareness were enhanced.

At the same time, teachers guided the students to participate in the research projects of teachers, encouraged students to declare innovative projects and research topics, and conducted self-employment guidance in the practical teaching base. So far, relying on the base, the students had applied for 4 patents, applied for 6 subjects, and published 15 papers.

RETRACTED

### 4.2. Beautifying the Campus and Creating a Campus Culture

According to the needs of the university landscape, the campus had been beautified and a comfortable environment for teachers and students had been created through such projects as planting flowers in tree pools, transforming *Prunus mume* forests and transforming *Cedrus deodara* forests [12]. Under the guidance of teachers, students listed plants on the campus and marked plant species and ecological habits, which could not only serve as the result of students' practical training but also provide reference for teachers and students of other majors to gain science knowledge, so that teachers and students could better care for the campus environment (Figure 6). At present, more than 80% of plant species on campus had been listed. Under the guidance of teachers, students took photographs and collected materials of plant species on campus and prepared to publish a book on plant Atlas of Xuzhou University of Technology.

### 4.3. Improvement in the Practical Ability of Professional Teachers

Professional teachers of landscape architecture majors learned and practiced at the base at any time, followed closely the new development of the landscape industry, and mastered the new knowledge and technology of landscape architecture in time. The professional practice ability had been exercised and the practice level of landscape architecture teachers had been improved and strengthened. At present, there were 11 professional teachers in the landscape architecture major and 7 teachers had the qualifications of practical teachers. Among them, 4 teachers had the titles of engineers and senior engineers. A well-structured “double-skilled” faculty team was initially formed.

## 5. Discussion and Conclusion

Our university made full use of the campus environment to exploratorily establish the campus practical teaching base for landscape architecture majors. This not only absorbed the theory of the production practical teaching base in higher vocational colleges but also applied it in applied undergraduate universities in combination with practice [13–16]. Our university constantly summarized and refined the combination of theory and practice, and in turn guided the construction of practical teaching bases and teaching reforms. The practical teaching base based on the campus environment had both scientific basis and practical test and realized the integration of theory and practice.

The establishment of the practical teaching base of landscape architecture majors in our campus aimed at cultivating students' practical innovation ability and improving teaching quality in a large area, while the “double-qualified” teachers training and teaching reform closely combined with the improvement of campus environmental quality, so as to the beneficial groups (including students, teachers, schools, etc.) were maximized with the construction of the practical teaching base.

RETRACTED

As the service department of the university, the logistics office has many of the resources that can be combined with the practical training of the university specialty, such as campus greening, power supply, water supply, and drainage. However, it remains a question as to how to combine the logistics resources and students' professional training effectively, so that the logistics resources can effectively serve the practical teaching of each major, and at the same time, each major makes full use of its own advantage to feed back in the logistics construction, which requires the joint efforts of multiple departments of the university. Under the overall planning of university leaders and the cooperation of various departments such as the secondary colleges, the student affairs office, the finance office, the equipment office, and the dean's office, the campus practical teaching base can not only save costs for the university but also serve the practical teaching of related majors, so as to achieve multiple integration and maximize the comprehensive benefits.

In future, the research on the campus practice teaching base can be conducted in depth from the aspects of the close degree of the combination of college majors and campus elements, students' practice and management methods, and the adjustment of talent cultivating programs.

## Figures and Tables

**Figure 1:** “Four in one” practical teaching base construction mode.

**Figure 2:** Cooperation mode of practical teaching base construction.

**Figure 3:** Management model of the campus's practical teaching base.

**Figure 4:** Landscape design competition works.

**Figure 5:** Plant pruning competition scene.

**Figure 6:** Campus beautification and culture construction.

**Table 1:** “Four-stage” progressive training teaching chain form.

Training stage	Training course	Schedule
Basic practical ability training stage	Cognitive practice, art sketch, surveying practice, landscape botany practice	Semesters 1–4

Professional core skills' training phase	Landscape architecture design practice, landscape planning and design practice, landscape engineering practice	Semesters 4–6
	Plant landscape design practice	

Comprehensive application ability training stage	Comprehensive practical training	Semesters 6–8
	Graduation design	

Innovation and entrepreneurship capacity training stage	Innovation and entrepreneurship quality education for university students	Semesters 2–8
	Graduation practice, innovation and entrepreneurship competition	

RETRACTED

## Data Availability

The datasets used and/or analyzed during the current study are available from the corresponding author on reasonable request.
